The article "Molecular mechanisms in progression of HPV-associated cervical carcinogenesis" was retracted in 2019. Reasons: plagiarism; overlap with other authors' work.

# Molecular mechanisms in progression of HPV-associated cervical carcinogenesis

**DOI:** 10.1186/s12929-019-0520-2

**Published:** 2019-04-23

**Authors:** Sadhana M. Gupta, Jayanti Mania-Pramanik

**Affiliations:** Department of Infectious Diseases Biology, National Institute for Research in Reproductive Health, J.M. Street, Parel, Mumbai, 400012 India

**Keywords:** Cervical carcinogenesis, Oncogene expression, Chromosomal mutations, Epigenetic alterations

## Abstract

Cervical cancer is the fourth most frequent cancer in women worldwide and a major cause of mortality in developing countries. Persistent infection with high-risk human papillomavirus (HPV) is a necessary cause for the development of cervical cancer. In addition, genetic and epigenetic alterations in host cell genes are crucial for progression of cervical precancerous lesions to invasive cancer. Although much progress has been made in understanding the life cycle of HPV and it’s role in the development of cervical cancer, there is still a critical need for accurate surveillance strategies and targeted therapeutic options to eradicate these cancers in patients. Given the widespread nature of HPV infection and the type specificity of currently available HPV vaccines, it is crucial that molecular details of the natural history of HPV infection as well as the biological activities of viral oncoproteins be elucidated. A better understanding of the mechanisms involved in oncogenesis can provide novel insights and opportunities for designing effective therapeutic approaches against HPV-associated malignancies. In this review, we briefly summarize epigenetic alterations and events that cause alterations in host genomes inducing cell cycle deregulation, aberrant proliferation and genomic instability contributing to tumorigenesis.

## Background

Cervical cancer is the fourth most frequent cancer in women with an estimated 5,70,000 new cases in 2018 representing 6.6% of all female cancers (WHO report, 2018). According to 2013 data from WHO, developing countries account for more than 85% of these cases. In India, the second most populous country in the world, over 80% of cervical cancers present at a fairly advanced stage. The current estimates in India indicate that every year 1,22,844 women are diagnosed with cervical cancer and 67,477 die from the disease (HPV and Related Cancers, Fact Sheet 2017). Infection with high risk human papillomavirus (HPV) has been recognized as an essential factor for the development of cervical cancer. HPV infection is the most common sexually transmitted infection worldwide and most sexually active individuals acquire it at some point of time during their life [1]. HPVs can also cause cancer of the vagina, vulva, penis, and anus, as well as some head and neck cancers, anogenital warts, and recurrent respiratory papillomatosis. Most HPV infections (~90%) clear within 6-18 months after acquisition, without any clinical signs or symptoms (transient infections) [2, 3]. However, some infections become persistent and increase the risk of premalignant or malignant disease [4]. Of these, only 0.3%–1.2% of initial infections will eventually progress to invasive cervical cancer. In addition to HPVs, other risk factors for progression to cervical cancer are immunodeficiencies such as in renal transplantation or human immunodeficiency virus disease [5], although sexual and reproductive factors, long term oral contraceptive use [6] smoking [7] and *Chlamydia trachomatis* infection [8] have also been implicated [4].

### Natural history of Human Papillomavirus (HPV) infection

Human papillomaviruses (HPV) are DNA tumor viruses belonging to the Papillomaviridae family. More than 200 human and animal papillomavirus genotypes have been characterized and sequenced. Of the approximately 30 HPVs that infect the anogenital tract, 15 HPV types, classified as ‘high-risk’ types (HPV types 16, 18, 31, 33, 35, 39, 45, 51, 52, 56, 58, 59, 68, 73 and 82) are associated with high grade lesions and invasive cervical cancer [9]. Of these, HPV16 and HPV18 are the most important types, causing ∼70% of squamous cell carcinomas, and >90% of adenocarcinomas [10]. On the other hand, 11 different HPV types, classified as ‘low-risk’ HPV types (HPV types 6, 11, 40, 42, 43, 44, 54, 61, 70, 81 and CP6108) are mainly associated with genital warts and benign cervical lesions. The human papillomaviruses are non-enveloped DNA viruses with icosahedral capsid that consists of a circular double stranded DNA 7900 bp long. According to protein expression during the viral cycle, two functional genome regions have been identified: (i) a coding region containing the early genes, E1, E2, E4, E5, E6, and E7 and (ii) a region containing two late genes, the major (L1) and minor (L2) capsid proteins. In addition, the HPV genome has a non-coding region, termed long control region (LCR), which includes most of the regulatory elements involved in viral DNA replication and transcription [11]. During HPV infection, the different viral proteins are expressed sequentially.

The present review focuses on understanding the etiology of HPV-mediated carcinogenesis, the cellular pathways and molecular mechanisms involved in transition from HPV infection to malignant transformation leading to cervical cancer.

## Main Text

### HPV Life cycle

The life cycle of HPV is intimately linked to the differentiation status of the host cell keratinocyte and is characterized by distinct phases of replication [12, 13]. High-risk and low-risk HPVs initiate infection by gaining access to the proliferating basal cells of the stratified epithelium through a micro abrasion [14] (Fig.1). The mechanisms allowing entry from the extracellular milieu into the cell are known to proceed through interaction with cell surface heparan sulphate followed by clathrin- or caveola-mediated endocytosis [15, 16]. During productive infection, the viral genome is maintained at a low copy number as an extrachromosomal element known as episome in the basal undifferentiated cells of the epithelium. HPV undergoes a transient round of replication referred to as “establishment replication”, which results in a copy number of 50–100 viral genomes per cell. These viral episomes are maintained in undifferentiated basal cells by replicating alongwith the host cell chromosomes. Thereafter, the viral life cycle is tightly coupled to the differentiation program of keratinocytes and relies on several cellular factors and viral proteins.

**Fig. 1:** Organization of HPV genome. **a.** HPV genome has a circular double-stranded DNA (8000bp). The viral genes are transcribed in a single direction (clockwise). There are genes coding for non-structural proteins (E1, E2, E4, E5, E6, and E7) and structural proteins (L1, L2), and a transcriptional control region (long control region; LCR). LCR contains a DNA replication origin and functions as a regulator for DNA replication. **b.** The HPV lifecycle. Human papillomavirus is thought to reach the basal cells through microabrasions in the cervical epithelium. After infection, the early human papillomavirus genes E1, E2, E4, E5, E6, and E7 are expressed and the viral DNA replicates from episomal DNA and establishes ∼50 HPV episome copies, which then segregate between the daughter progeny as the cells undergo cell division. In the upper layers of epithelium, viral genome is replicated further, and late genes L1 and L2, and E4 are expressed. The early viral proteins E6 and E7 are key to stimulating proliferation and milieu for E1 and E2-driven viral genome replication to a high copy number. Integration of human papillomavirus genome into the host chromosome occurs with associated loss or disruption of E2, and subsequent upregulation of E6 and E7 oncogene expression. Terminal differentiation of infected cells in the upper epithelial layers activates the expression of E4 and then L1 and L2 to encapsidate the viral genomes to form progeny virions. The shed virus can then initiate a new infection

The replication of viral genome requires the viral initiator protein E1, which contains a helicase-ATPase activity, and the multifunctional viral protein E2, which helps in the specific recruitment of E1 to the viral DNA. E1 oligomerizes and assembles as a double-hexamer at the viral origin of DNA replication and functionally interacts with several host replication factors, such as polymerase α-primase, replication protein A, topoisomerase I and cyclin E/Cdk2 [17]. E2 also functions as a transcription factor, capable of trans-activation and repression [18] and as a mediator of genome segregation, which is essential for viral persistence [19]. As the infected cells undergo differentiation, late gene expression and viral genome replication are induced. E4 and E5 are both required for viral amplification. To maintain the cellular replication machinery active, the viral proteins E6 and E7 are expressed and uncouple cell growth arrest and differentiation primarily through the inactivation of p53 and pRb, respectively. The inactivation of pRb by E7 forces infected cells to remain in a proliferative state and escape cell cycle exit, while abrogation of p53 by E6 ensures cell survival by preventing apoptosis triggered by this aberrant growth signal. The productive phase of the viral life cycle is activated further upon epithelial differentiation, resulting in the amplification of viral genomes to thousands of viral copies per cell in the suprabasal layers, as well as activation of late gene expression [13, 20]. The amplified genomes are then packaged into infectious virions by the L1 and L2 proteins, which form the subunits of the icosahedral capsid. Finally, viral escape probably occurs by natural tissue desquamation and may be facilitated by the keratin network disrupting ability of E4 [21].

The regulation of viral life cycle in this manner allows HPV to avoid detection by the immune response as high levels of viral gene expression as well as virion production are restricted to the uppermost layers of the epithelium, which are not under immune surveillance [22]. Due to small coding capacity of the viral genome, HPV depends on the host DNA replication machinery to synthesize its DNA. In order to support productive replication, HPV employs numerous mechanisms to subvert key regulatory pathways that regulate host cell replication, maintaining the differentiating cells active in the cell cycle. As such, HPV is able to reactivate cellular genes and signalling pathways necessary to support late gene expression and amplification of viral DNA.

### Molecular events in cervical cancer progression

A complex network of interactions involving various factors are important for transformation and malignant progression. Cervical carcinogenesis is a multistage process associated with the accumulation of DNA alterations in host cell genes. These alterations involve both epigenetic and genetic changes in oncogenes and tumour suppressor genes which are crucial regulators of cell cycle progression, chromosomal stability, telomere activation and apoptosis. But the pivotal step for the onset of tumorigenesis appears to be the integration of viral genome into the host.

### HPV Integration and overexpression of oncogenes E6/E7

Integration of HPV DNA into the host cell genome is a key event in HPV-mediated carcinogenesis leading to aberrant proliferation and malignant progression [23, 24]. Integration impacts the host genome by amplification of oncogenes and disruption of tumor suppressor genes as well as driving inter- and intra-chromosomal rearrangements [25].

The early genes E6 and E7 play an essential role in HPV-induced carcinogenesis by interfering with two essential tumor suppressor genes p53 and pRb that regulate normal cellular proliferation. The interaction of Е7 with pRb protein causes its degradation and aberrant initiation of S-phase and release of E2F transcription factor that triggers the expression of cyclins and other S-phase regulators. The mechanism of Е6/Е7-induced transformation is not confined exclusively to the degradation of the key cellular “guardians” pRb and р53. E7 also associates with other proteins involved in cell proliferation, including histone deacetylases [13], components of the AP1 transcription complex [26] and the cyclin-dependent kinase inhibitors p21 and p27 [27]. At the same time, Е6 protein targets р53 for proteasomal degradation and causes inhibition of apoptosis and DNA repair which is an integral component of the HPV life cycle. The degradation of p53 by E6 is important because p53 is a transcription factor that regulates the expression of genes encoding regulators of cell cycle, DNA repair machinery, metabolism and apoptosis [21]. This is of key importance in the development of cervical cancers, as it compromises the effectiveness of cellular DNA damage response and allows the accumulation of secondary mutations.

Recent studies indicate the existence of an intricate HPV interactome, i.e., a network of intermolecular interactions of Е6 and Е7 with the host cell proteins [28]. By these interactions, the Е6 and Е7 proteins can modulate the profile of gene expression, host cell proteome, and intracellular signaling pathways (including MAPK-, Wnt-, Akt-, Notch-, mTORC-, and STAT-dependent cascades), leading to remodelling of epithelial cells [29]. In addition, E6 also binds to and degrades FAS-associated death domain protein (FADD), preventing the transmission of apoptotic signals via the Fas pathway [30]. All these molecular alterations facilitate resistance to programmed cell death, or apoptosis. Apoptotic cell death also requires the involvement of caspases which are key molecular players of the apoptosis regulatory network [31]. Thus, the continuous activity of E6 and E7 proteins leads to aberrant cell proliferation, accumulation of oncogene mutations, and ultimately cervical cancer.

### Molecular mechanism of HPV integration and overexpression of E6/E7 oncoproteins

Integration typically results in the increased expression and stability of transcripts encoding the viral oncogenes E6 and E7, which are known to inactivate and/or accelerate the degradation of numerous cellular proteins, including retinoblastoma protein (E7) and p53 (E6) [32]. The site of integration is distributed throughout the genome as chromosomal fragile sites where DNA double strand breaks fail to repair and FRA8C at chromosome 8q24 near the c-myc locus has been reported as one such example [33]. Integration starts with DNA damage, induced either by oxidative stress or HPV protein and the subsequent steps are driven by the DNA damage responses (Fig. 2). Breaks in HPV DNA are introduced during the replication of virus and these breaks fail to get repaired. HPV takes advantage of this damage response pathway for its own replication and produces an adequate number of episomal HPV which increase the availability of more HPV DNA for integration into the host DNA. The DNA break-induced DNA damage response (DDR) triggers the accumulation of factors for replication at the replication foci and acts as a driving force throughout viral replication [34]. Virus uses the DDR machinery to promote viral amplification while the viral oncoproteins render the cells to overcome the downstream consequences of damage response. The oncoproteins E6 and E7 disrupt cell cycle checkpoint control by inhibiting CDKs inhibitors (P21, P27) and degrading P53 [13]. HPV-16 E7 oncoprotein attenuates the DNA damage checkpoint response by accelerating the proteolytic turnover of claspin, a critical regulator of the ATR/CHK1 signaling axis and DNA damage checkpoint recovery in G2 phase of the cell cycle [35]. In addition, proximity between viral and host genome by E2-BRD4-mediated tethering could increase the feasibility of viral integration. The fusion between both the genome via either homologous or nonhomologous recombination is regulated by the DNA damage response pathway (ATM/ATR and DNA-PK pathways) [36].

**Fig. 2:** Mechanism of HPV DNA integration: Induction of double strand breaks by reactive oxygen species, viral protein induces DNA damage response, following which ATR and P53 get activated to repair the damage. HPV oncogenes deactivate the normal function of DNA damage response (DDR). E7 acts on ATR and degrades claspin, inactivates Rb disrupting the cell cycle inhibitors p21, p27. E6 degrades p53 inhibiting DNA repair, degrades FAS-associated death domain protein (FADD) preventing apoptosis via Fas pathway, promotes degradation of transcriptional repressor, NFX1 and activates hTERT transcription. Virus utilizes the DDR machinery for its replication and close proximity with host genome is mediated by the Bromodomain protein 4, BRD4-E2 complex. The fusion between host and viral genome is accomplished by Nonhomologous mediated end joining (NHEJ) finally leading to integration of HPV DNA into the host genome

The association of head-to-tail tandem repeats in the chromosome of cervical cancer cells [37] indicates that a linear concatemeric HPV genome is synthesized by a rolling circle mechanism of replication which integrates into the host chromosome [38]. It has been reported that homologous recombination machinery recruited to the regions of double strand breaks only is generated through collapsed replication fork during replication of viral genome [39]. In addition, HPV genome tethers to host chromatin by HPVE2-BRD4 (Bromodomain protein 4) complex for partitioning of genomes to daughter cells [40]. The association of BRD4 with the chromosomal fragile region suggests that BRD4 may play an important role in increasing the mechanistic feasibility of integration. Finally, the loss of E2 ORF during integration causing enhanced expression of viral oncogenes E6 and E7, leading to disruption of critical cellular genes plays an important role in progression to carcinogenesis.

### Chromosomal alterations

The viral oncoproteins E6 and E7 are known to induce DNA damage, centrosome abnormalities and chromosomal segregation defects, thereby leading to chromosomal instability [41, 42]. High-risk E6 has the ability to activate the catalytic subunit of telomerase [hTERT (human telomerase reverse transcriptase)], which adds hexamer repeats to the telomeric ends of chromosomes [43]. HPV16 E6 associates with E6AP, to promote the degradation of the transcriptional repressor NFX1-91, and consequently activate hTERT transcription; this repressor has also a role in HPV16 E6 activation of the oncogenic transcription factor NF-ҡB [44]. HPV infected cells display a very high level of telomerase activity, allowing telomere length maintenance and indefinite proliferation [45]. The activity of telomerase is normally restricted to the proliferative compartment of epithelium, and activation is associated with cellular immortalization and carcinogenesis [46].

It has been reported that, several regions are typically lost in cervical carcinogenesis (2q, 3p, 4p, 5q, 6q, 11q, 13q and 18q) while other regions are amplified (1q, 3q, 5p and 8q) [47]. The 3q26 region contains sequences for the RNA component of human telomerase gene, which serves as a template for addition of telomeres, which is the basis for telomerase based cell immortalization [48]. The frequency of 3q26 gain has been found to increase with the severity of cervical neoplasia [49].

### Epigenetic changes

In addition to genetic alterations, it has become evident that oncogenomic processes can be profoundly influenced by epigenetic mechanisms. Epigenetic alterations are often found early in tumorigenesis and are likely to be key initiating events in certain cancers [50]. In addition to tumor initiation, epigenetic events also contribute to tumor progression [51]. A number of epigenetic alterations have been identified that occur in both the HPV and the cellular genome, including DNA hypomethylation, hypermethylation of tumor suppressor genes, histone modifications, and alterations in ncRNAs.

### DNA methylation

The earliest and most common molecular changes in the multistep carcinogenesis process is DNA methylation [52]. In normal cells, DNA methylation is involved in the regulation of gene expression, including chromatin organization and genomic imprinting [53]. In contrast, global DNA hypomethylation in repetitive regions and hypermethylation in CpG islands of tumor suppressor gene promoters are observed in tumors [54, 55], and increase in the activity of (DNA methyltransferases (DNMT) 1 [56]. These alterations are also observed in HPV-induced carcinogenesis. HPV E7 binds to DNMT1 and stimulates its activity [57], and activates transcription of DNMT1 through the pRB/E2F pathway [58], while HPV E6 upregulates DNMT1 by suppression of p53 [59]. Increased expression of DNMT3A and 3B has also been observed in HPV-positive cells [60–62]. Aberrant methylation occurs frequently in cervical cancer, leading to silencing of gene expression, activation of oncogenes and transposable elements, loss of imprinting, and inactivation of tumor suppressor genes [63]. The activities of E6 and E7 causing increase in activity of DNMT1 results in hypermethylation of tumor-suppressor gene promoters, leading to silencing of genes (Fig. 3).

**Fig. 3:** Schematic presentation of DNA methylation by E6 and E7 oncoproteins: Binding of E6-E6AP complex to p53 to leads to ubiquitination and degradation of p53 and induces overexpression and activity of DNA methyltransferase (DNMT) 1. Binding of E7 to pRb causes the release of E2F, favoring the overexpression of DNMT1. The activities of E6 and E7 causing increase in activity of DNMT1 results in hypermethylation of tumor-suppressor gene promoters, leading to silencing of genes, cellular transformation and tumorigenesis

Various studies have found that methylation of CpG islands within the promoter regions of tumor suppressor genes can lead to silencing of gene expression. Epigenetic silencing of tumor suppressor genes plays an important role in cervical carcinogenesis [54]. This is an important epigenetic mechanism, tends to accumulate with disease severity [64, 65] and has been demonstrated in cervical cancer and its precursors [63]. A wide range of host genes involved in cell cycle regulation, apoptosis, DNA repair and WNT pathway often undergo epigenetic modification in cervical cancer.

The most frequently methylated genes in cervical cancer are cell adhesion molecule 1 (CADM1), Cyclin A1(CCNA1), cadherin 1 (CDH1), death-associated protein kinase 1 (DAPK1), Erythrocyte membrane protein band 4.1 like 3 (EPB41L3), myelin and lymphocyte (MAL), paired box 1 (PAX1), PR domain containing 14 (PRDM14,) and telomerase reverse transcriptase (hTERT) [64, 66–69]. Ras association domain family member 1(RASSF1), a key gene involved in the apoptotic signaling pathway is downregulated in cervical cancer via methylation [70]. Another study indicated that tumor suppressor gene CADM1 gene is silenced in cervical cancer due to methylation of the promoter region [71]. Downregulation of CADM1 gene leads to metastasis and cancer progression. Promoter hypermethylation is associated with decreased expression of CADM1 in high grade CIN and SCC [72]. Another gene CDH1 is downregulated due to promoter methylation in HPV positive cervical cancer [73]. A recent study showed that PRDM14 is downregulated in cervical cancer HPV positive cell lines due to promoter hypermethylation and its abnormal levels resulted in apoptosis [74]. A pro-apoptotic serine/threonine kinase, DAPK which plays a major role in metastasis and tumour pathogenesis [75] is reported to be inactivated due to hypermethylation in cervical cancer [76, 77]. Furthermore, methylation of decoy receptors (DcR1 and DcR2) was reported in HPV related cervical cancer leading to silencing and inhibition of apoptosis [78].

The silencing of E6 and E7 was found to decrease methylation of tumour suppressor genes and reverse the transformed phenotype of cervical cancer cells [61, 63]. Methylation of HPV genes with concomitant silencing of HPV oncogenes could be a strategy of the virus to maintain a long-term infection by evading immune recognition [79]. Several studies have shown that the frequency of DNA methylation of candidate genes increases with increasing severity of the cervical lesion, suggesting that these changes occur early in cancer development [64, 69, 80, 81]. Methylation is found to be more common in invasive cervical carcinoma and cervical intraepithelial neoplasia (CIN) III than in CIN I-II (84.6% and 46.2% vs. 29.4%, respectively) as reported by Hong et al. in 2008 [82]. Increased methylation levels at multiple CpG (Cytosine phosphate Guanine) sites have been reported in the E2, L2 and L1 regions in women with CIN3 and found to be greater than those in women with transient infections [83]. These epigenetic alterations in HPV infected host cells could serve as molecular markers of malignant transformation.

### Histone modifications

In addition to DNA methylation, the epigenetic regulation of gene expression is also impacted by histone modifications and the remodeling of nucleosomes. Histones can undergo a variety of post-translational modifications at the N terminus, which is represented by acetylation, methylation, phosphorylation, sumoylation, ADP–ribosylation, and ubiquitination. They can alter the DNA histone interaction, with a major impact on chromatin structure [84]. Distinct posttranslational modifications on histones, characterize transcriptionally active and silent chromatin

One mechanism by which HPV E6 and E7 oncoproteins alter the transcriptional competence of infected cells is by associating with and/or modulating the expression, as well as activities, of histone-modifying and chromatin-remodeling enzymes (Fig. 4). For example, acetylation of lysine residues of histones 3 and 4 (H3 and H4) by Histone acetyl transferases (HATs) leads to transcriptionally active chromatin, while the removal of these marks by Histone deacetylases (HDACs) results in transcriptionally repressed chromatin [85, 86]. The balance between activity of these enzymes has a key role in regulating gene transcription. E6, E7 oncoproteins can associate with enzymes that modulate histone acetylation, and thus, regulate the transcriptional capacity of host cell chromatin [85]. E6 high risk HPV protein shares with other DNA tumorigenic viruses the ability to target CBP/p300. Both HPV E6 and E7 can associate with and modulate the activity of the HATs p300 and CBP [87]. p300/CBP regulates a number of genes [88, 89]. HPV E6 inhibits p300/CBP-mediated acetylation of p53 [90] while HPV E7 forms a complex with p300/CBP and pRb, acetylating pRb and decreasing p300/CBP levels [91]. HPV E7 also associates with p300/CBP-Associated Factor (pCAF), reducing its ability to acetylate histones [92] and the steroid-receptor coactivator (SRC1), and abrogating SRC1-associated HAT activity [93]. Thus, E6, E7 protein binding to the transcriptional co-activator p300/CBP is a crucial step in cellular transformation.

**Fig. 4:** Schematic presentation of Histone modifications by HPV E6 and E7 interaction with cellular epigenetic modifiers. HPV oncoproteins E6, E7 bind to and/or modulate the expression of histone modifying enzymes, class I Histone deacetylases (HDAC), Histone acetyltransferases (HATs), Histone lysine demethylases (KDMs) and subunits of chromatin remodeling complexes. These interactions contribute to chromatin remodelling and transcriptional regulation leading to either activation or repression of gene expression

The HPV E7 oncoprotein interacts with class I HDACs [85], which function as transcriptional co-repressors by inducing chromatin remodeling via the reversal of acetyl modifications on histone lysine residues. The association of E7 and HDAC1/2 occurs in an Rb-independent manner through the intermediary Mi2β, a member of the nucleosome remodeling and histone deactylation (NuRD) complex; the NuRD complex remodels chromatin structure through the deactylation of histones and ATP-dependent nucleosome repositioning [94]. The association of E7 and HDAC1/2 plays a role in HPV E7-associated transcriptional regulation. Furthermore, HPV E7 can interact with interferon response factor 1 (IRF1) and recruit HDACs to suppress IRF1 transcriptional activity [95]. HDAC function is also necessary for HIF-1 (hypoxia inducible factor-1) activity, and it was found that E7HPV protein can block the interaction of HDACs with HIF-1α, activating HIF-1-dependent transcription for a range of pro-angiogenic factors [96]. Silencing of proliferation repressor protein osteo-protegerin (OPG) and retinoic acid receptor β2 (RAR-β2) was found to occur through histone modification as well as DNA methylation [97, 98].

The oncoproteins E6 and E7 are also involved in histone methylation which is acknowledged to be a dynamically controlled process by two types of enzymes that work together to maintain global histone methylation patterns- Histone methyl transferases (HMTs) and histone lysine demethylases (KDMs) [99]. Histone methylation may occur on different lysine residues and the interplay between HMTs and KDMs regulates the methylation level and contributes to the activation or repression of gene expression, depending on the specific lysine residue on which they act. Especially, KDMs expression has been found to be deregulated and associated with cancer aggressiveness. McLaughlin-Drubin et al [86] sustain that E7 HPV16 can induce epigenetic and transcriptional alterations by transcriptional induction of KDM6A and KDM6B histone 3 lysine 27 (H3K27)-specific demethylases. In addition, KDM5C demethylase is recruited by the E2 viral protein for E6 and E7 oncogenes transcriptional repression through the LCR region of HPV. KDM5C expression levels were found to be increased in CIN2+ lesions and significantly increased in SCC cases [100].

It is reported that, HPV modulates the activity of two coactivator histone arginine methyltransferases, CARM1 and PRMT1 leading to histone methylation on arginine residues. HPV E6 downregulates their expression, and these HMTs are needed for HPV E6 to attenuate p53 transactivation. E6 hinders CARM1- and PRMT1-mediated histone methylation at p53-responsive promoters and suppresses p53 binding to DNA [101]. E6 also inhibits SET7, which, in addition to catalyzing H3K4 monomethylation, methylates non-histone proteins, including p53 and downregulates p53K372 mono-methylation, thereby reducing p53 stability [102]. Together, the modulation of CARM1, PRMT1, and SET7 provides another mechanism by which HPV alters p53 function. There is a strong interplay between DNA hypermethylation and histone deacetylation for silencing and modulating the expression of a number of cancer-related genes that predicts not only a synergy in gene expression at global and individual gene levels but also in antitumor activity.

### Aberrant expression of non coding RNAs

Aberrant expression of non-coding RNAs, such as Long non coding RNAs (lncRNAs) and microRNAs (miRNAs) has been reported to play a vital role in the progression of cervical cancer.

- Long non coding RNAs (LncRNAs)

LncRNAs are long non coding RNAs involved in many diverse biological processes [103, 104]. Altered expression of lncRNAs is specifically associated with tumorigenesis, tumor progression and metastasis. Several lncRNAs have been found to be aberrantly expressed in cervical cancer. Hox transcript antisense intergenic lncRNA (HOTAIR), a long intergenic ncRNA (lincRNA) was found to be increased in cervical cancer tissues and correlated with FIGO stage, lymphatic metastasis, tumor size and invasive depth, indicating its involvement in cervical cancer progression [105]. It has also been reported that, HOTAIR might accelerate neoplasm aggressiveness by upregulation of VEGF, MMP-9, and epithelial-mesenchymal transition (EMT)-related genes by decreasing the expression of E-cadherin while increasing the expression of β-catenin, Vimentin (VIM), Snail, and Twist [106]. Sharma et al reported that the crosstalk between HPV16 E7 oncoprotein and lncRNA HOTAIR was concomitant with cellular proliferation and metastasis in cervical cancer [107].

A few lncRNAs, were found to be downregulated namely growth arrest-specific transcript 5 (GAS5), Tumor suppressor candidate 8 (TUSC8) and lncRNA low expression in tumor (lncRNA-LET). GAS5 was downregulated in cervical cancer tissues and significantly correlated to advanced cancer progression [108]. TUSC8 plays pivotal role in cell proliferation through downregulating c-Myc level in cervical cancer. The expression of TUSC8 was significantly decreased in cervical cancer and linked to FIGO stage, size of tumor, and squamous cell carcinoma antigen [109]. LncRNA LET, a newly identified lncRNA, was found to be downregulated in hepatocellular carcinomas, colorectal cancers, squamous cell lung carcinomas, and cervical cancer [110].

(b) micro RNAs (miRNAs)

Besides protein coding genes, methylation mediated silencing of non-coding microRNAs (miRNAs) has also been detected in cervical lesions [111]. MicroRNAs(miRNAs) are short non-coding RNAs regulating cellular processes such as cell proliferation, cell cycle progression, apoptosis, and metastasis. The expression of viral oncoproteins can modulate the expression levels of miRNAs enhancing malignant progression leading to invasive cancer. HPVs modulate the expression of host miRNAs [112] via deletion, amplification, or genomic rearrangement. Complex interactions between HR-HPV E6 and E7 involve the activation of transcription factors, such as E2F and c-Myc, which can promote the transactivation of miRNAs [113]. Continuous E6/E7 expression is linked to a decrease in the intracellular concentrations of miR-23a, miR-23b, miR-27b, and miR-143, all linked to anti-tumorigenic activities [114].

The carcinogenesis process is influenced by up regulation as well as down regulation of miRNAs. Increased expression of certain mi-RNAs (viz., miR-886-5p, miR-10a, miR-141, miR-21, miR-135b, miR-148a, miR-214 and miR-106b) plays vital role in cervical cancer progression as they are involved in regulation of cell proliferation, apoptotic pathway or cell adhesion [115, 116]. Zheng et al found that the expression level of miR-31 was significantly higher in cervical cancer patients than in normal individuals [117] and the expression of HPV16 E6/E7 oncoproteins increased miR-31 levels. Furthermore, they reported that the overexpression of miR-31 can promote cell proliferation and enhance the migration and invasion abilities of cervical cancer cells. Liu et al observed that miR-9 was upregulated in HR-HPV-positive tumors by both E6 and E7 oncoproteins, and that activation of this miRNA by HPV E6 oncoprotein was independent of the p53 pathway [118]. Furthermore, overexpression of miRNA-21 has been associated with aggressive progression and poor prognosis in cervical cancer [119]. MiR-21 is transcriptionally induced by Activator Protein 1 (AP-1) which is essential for HPV transcription.

The down regulation of let-7c, miR-124, miR-126, miR-143, and miR-145 has been found to regulate the expression of oncogenes. MiR-34a has been identified as a direct transcriptional target of cellular transcription factor p53 [120]. As HPV E6 oncoprotein destabilizes p53 during oncogenic HPV infection, a down-regulation of miR-34a expression is observed. MiR-34a targets multiple cell cycle components, including CDK4, cyclin E2, E2F-1, hepatocyte growth factor receptor MET, and Bcl-2 [121, 122]. Melar-New and Laimins recently demonstrated that E7 protein has the ability to downregulate miR-203 expression upon differentiation, which may occur through the mitogen-activated protein (MAP) kinase/protein kinase C (PKC) pathway [123]. Hence, it is conceivable that, expression of E6 and E7 can modulate expression levels of miRNAs, enhancing the progressive alterations leading to invasive cancer.

### Structure - based function studies of E6 and E7 proteins

#### HPV E6

The full-length oncoprotein E6 is a basic nuclear protein (~18 kDa) composed of approximately 150 amino acid residues. Similar to E6 proteins encoded by other papillomaviruses, the 16E6 contains four zinc-binding motifs (Cys-X-X-Cys) and forms two Cys/Cys fingers that bind zinc directly [124]. These motifs are strictly conserved in all E6 proteins and their integrity is essential for the oncoprotein’s normal functions. 16E6 also contains a PDZ domain–binding motif at its C-terminal extremity [125, 126] and three nuclear localization signals (NLSs) (Fig. 5). PDZ domains are approximately 90 amino acid protein-protein interaction domains [127]. HPV-16 and HPV-18, are known to interact with numerous PDZ-domain containing proteins via their PDZ-binding motifs [128]. These are involved in the regulation of epithelial cellular polarity, emphasizing the importance of this pathway for viral replication and HPV-driven malignancy. The PDZ-binding motif is also important in viral life cycle, since its loss reduces viral replicative potential and leads to episomal integration [129, 130].

**Fig. 5:** Schematic structure of oncoprotein E6. Protein structure and functions of HPV16 E6. Four zinc-binding motifs are indicated as grey boxes. The two zinc fingers are shown together with regions that are involved in interacting with some of its cellular target proteins. E6 contains PDZ domain–binding motif at its C-terminal extremity and three Nuclear localization signals (NLS). Functions associated with proteins in different regions are indicated by arrows

The crystal structures of both N-terminal and C-terminal halves, as well as the complete structure of the E6 proteins [131] have confirmed the fact that E6 interacts with a wide range of cellular substrates [132]. The principal cellular target of HR E6 proteins is the tumor suppressor p53. High-risk E6 interacts with E6AP and tumor suppressor protein p53 to induce ubiquitination-mediated degradation of p53 [133]. E6 hijacks a cellular E3 ubiquitin ligase UBE3A/E6AP (E6-associated protein), binding through E6’s LXXLL motif, and the stable E6/E6AP complex then labels p53 for degradation in a proteasome-dependent manner [134] Studies have shown E6 to be closely associated with other components of the proteasome degradation pathway: the E3 ubiquitin ligases UBR5/EDD and HERC2 [135]. Under hypoxic conditions, high-risk E6 also inactivates the CYLD tumor suppressor through interactions with CYLD deubiquitinase to allow unrestricted activation of NF-κB [136].

High risk E6 oncoproteins are also involved in the deregulation of cellular DNA replication machinery. Besides the ability to immortalize and transform cells and induce p53 degradation, 16E6 is known to be functionally involved in regulating gene transcription [137]. 16E6 can interact with other transcription factors and coactivators, including p300/CBP [133], IRF-3 [138] and c-Myc [139]. HPV-16 E6 induces telomerase activity in primary epithelial cells through transcriptional transactivation of the hTERT telomerase catalytic subunit [41, 140]. The 16E6–c-Myc interaction induces transcription of h-TERT to promote cell immortalization [141]. Furthermore, it has been demonstrated that E6-interacting regions of p300 are necessary for E6 to inhibit p53-dependent chromatin transcription. E6-mediated repression of p53 correlates with inhibition of acetylation on p53 and nucleosomal core histones, altering p53 and p300 recruitment to chromatin [90].

In addition, 16E6 is an RNA binding protein and interacts with cellular splicing factors and RNA via its C-terminal NLS3 to regulate splicing of E6E7 bicistronic RNAs [142]. The multifunctional activity of 16E6 is not restricted to the nucleus, because it can act as a regulator of signal transduction through interacting with cytoplasmic E6BP (Erc55) [143], protein tyrosine phosphatase H1 [144] and PDZ proteins such as SAP97/hDlg [145]. All HR HPV E6 proteins have a class I PDZ (PSD95/Dlg/ZO-1)-binding motif (x-T/S-x-L/V [146] at their C-termini. Thus, these interactions suggest that 16E6 and other high-risk E6s can be regarded as multifaceted viral proteins with characteristic and distinct activities in the nucleus and cytoplasm of the cells they infect.

#### HPV E7

The full-length oncoprotein E7 is a nuclear protein containing approximately 100 aa residues that has a C-terminal zinc-binding domain, whose structural integrity is critical for E7 activity [147]. E7 is post-transcriptionally regulated by the proteasome and by phosphorylation. The N-terminus of E7 contains sequence similarity to a portion of CR1 and the entire CR2 of adenovirus E1A and related sequences in SV40 T antigen. The CR2 region of E7 contains the CKII phosphorylation site and the LXCXE binding motif involved in binding to proteins such as the retinoblastoma tumor suppressor (pRb) (Fig.6). E7 uses its LXCXE motif to target unphosphorylated pRb for degradation via the ubiquitin proteasome pathway [148]. Oncogenic E7 induces the degradation of pRb by interacting with the cullin 2 ubiquitin ligase complex [149]. It has been also demonstrated that Casein Kinase II (CKII) phosphorylation of the E7 N-terminal domain is critical for its transformational activity and for its ability to drive S-phase progression [150]. The C-terminus of E7 may also be involved in zinc-binding [151].

**Fig. 6:** Schematic structure of oncoprotein E7. Protein structure and functions of HPV16 E7 and the most important amino acid motifs required for integrity and protein functions. Relative locations of the regions with sequence motifs similar to a portion of conserved region 1 (CR1) and the entire CR2 of adenovirus E1A are shown with the pRB-binding site LXCXE in the CR2. Zinc binding motifs are indicated in grey boxes. The zinc finger is shown together with the regions involved in pRb binding (LXCXE) and the two serine residues (31 and 32) that are susceptible to casein kinase II (CKII) phosphorylation. Functions associated with proteins in different regions are indicated by PI3K

High-risk E7 interacts with the pRb tumor suppressor protein via the LXCXE motif in the E7 CR2 domain to promote cell cycle progression [148]. Interaction with pocket proteins has been characterized as one of the major functions of E7. Oncogenic E7 binds related pocket proteins p107 and p130 with high affinity via the LXCXE motif in CR2, whereas low-risk or non-oncogenic E7 binds pRb with much lower efficiency. These play important roles in the regulation of cellular proliferation, differentiation and apoptosis. They inhibit E2F-mediated transcription and negatively regulate the transitions from G0 to G1, and into S phase of the cell cycle [152]. The LXCXE motif of the E7 CR2 domain that has been shown to be required for pRb inactivation is also required for down-regulation of p107 and p130 [153]. This indicates the necessity for interaction of E7 with the pocket proteins for its optimal ability to continually drive cell cycle progression. Among other binding partners that interact with this domain of E7 are UBR4/p600 [154] and p300/CBP-associated factor (P/CAF). Interaction between E7 and UBR4/p600 is required for E7-mediated cell transformation [155]. In addition to its main role in driving cell cycle progression, the interactions with substrates also indicate that E7 has a crucial role in destabilizing transcriptional complexes and in chromatin remodeling, consequently having an impact on cellular proliferation.

E7 contains a nuclear localization signal in the N-terminal domain (aa 1-37) [156]. In addition to its cellular transformation activities, oncogenic E7 also plays a role in the viral life cycle [157] and affects many other cellular activities in HPV-infected cells. E7 dysregulates the cell cycle by stabilizing p21 [158] and upregulating p16 expression [159]. Oncogenic E7 induces mitotic defects and aneuploidy by inducing centrosome abnormalities through its association with the centrosomal regulator γ-tubulin; this inhibits γ-tubulin recruitment to the centrosome [160] and leads to chromosomal instability. Thus the interaction of high-risk E6 and E7 with cellular tumor suppressor proteins and perturbation of normal cell cycle control are believed to be the most important factors for malignant conversion.

### Interaction of pathways in progression to cervical cancer

A coordinated interaction of multiple processes and signalling pathways is required for progression to oncogenesis (Fig.7). Multiple processes and signaling pathways are altered by HR-HPV E6 and E7 oncoproteins in cervical carcinogenesis [161] among other affected processes, genomic instability plays a central role leading to mutations in cellular genes, which cooperate with the initial necessary steps induced by HR-HPV oncoproteins, including inactivation of two important tumor suppressor pathways (pRB and p53). As mentioned earlier, E6 is able to induce the degradation of p53 via direct binding to the ubiquitin ligase E6AP, inhibiting p53-dependent signaling upon stress stimuli, and contributing to tumorigenesis. On the other hand, oncoprotein E7 associates with the retinoblastoma family of proteins (pRb, p107 and p130) and disrupts their association with the E2F family of transcription factors, subsequently transactivating cellular proteins required for cellular and viral DNA replication.

**Fig. 7:** Molecular events in progression to cervical carcinogenesis. Persistent infection with high risk HPV leads to integration of HPV into the host genome, leading to overexpression of oncogenes E6 And E7. Interaction of Е7 with pRb protein leads to aberrant initiation of S-phase, release of E2F transcription factor that triggers the expression of cyclins and CDK inhibitors p21 and p27, altering the integrity of cell cycle thereby contributing to cellular immortalization and transformation. Е6 targets р53 for proteasomal degradation leading to inhibition of apoptosis and DNA repair. E6 activates PI3K/Akt pathway, interacts with cellular proteins NFX1 and induces activation of hTERT leading to immortalization and transformation. The interaction of both onoproteins with DNMTs leads to aberrant methylation causing silencing of tumor suppressor genes. E7 interaction with HDACs causes chromosome remodeling and genome instability. Thus, the cross interaction of E6 and E7 with various pathways plays a key role in progression to carcinogenesis

The interaction of E6 with various pathways is associated with cancer initiation, progression and metastasis. Several studies indicate that E6 can activate PI3K/Akt pathway through various mechanisms. E6 inactivates PTEN through PDZ proteins, leading to increased pAkt as well as increased cell proliferation [162]. In addition, mammalian target of rapamycin (mTOR) a downstream target of Akt is activated by E6 as indicated by increased ribosomal protein S6 kinase [163]. The mTOR kinase is also activated by mitogen-activated protein kinase (MAPK) pathway. Activation of Akt can produce a cascade of changes in downstream targets. Akt can phosphorylate E6 to promote its ability to interact with protein 14-3-3σ, which is important in carcinogenesis [164]. HPV has also been associated with increased expression of c-myc, a downstream protein of Akt [165]. E6 has been reported to act directly on c-myc, leading to activation of telomerase activity [166]. Telomerase activation is critical for the immortalization of primary human keratinocytes by the high-risk HPV E6 [52]. E6 is able to increase telomerase activity by upregulation of telomerase reverse transcriptase (TERT), which is encoded by the human telomerase reverse transcriptase (hTERT) gene. E6 induces the hTERT promoter via interactions with the cellular ubiquitin ligase, E6AP. E6 increases hTERT via NFX1-123. NFX1-123 interacts with hTERT mRNA and stabilizes it, leading to greater telomerase expression [167]. Several studies have shown that E7 can also activate the PI3K/Akt pathway. The ability of E7 to increase Akt activity is correlated with its ability to bind to and inactivate Rb. Second, silencing of Rb by short hairpin RNAs (shRNAs) in differentiated keratinocytes leads to increased Akt activity. Third, increased Akt activity and loss of Rb were also correlated in HPV-positive cervical high-grade squamous intraepithelial lesions [168].

Activation of the Wnt/β-catenin, Notch and Hedgehog signaling pathways is characteristic of the cancer stem cells [169]. Recently, it has been found that Wnt/β-catenin signaling is a very important pathway in the maintenance of CSCs [170]. Lichtig et al [171] also showed that HPV16 E6 activated the Wnt/β-catenin pathway; the mechanism is independent of the ability of E6 to target p53 for degradation or bind to the PDZ-containing proteins. It has been demonstrated that, HPV16-associated cervical tumorigenesis is synergized by GSK3β inactivation and overactivation of the Wnt/β-catenin pathway [172]. Activation of the Wnt pathway results in accumulation of β-catenin, which in turn increases transcription of a broad range of genes to promote cell proliferation. Although the Wnt pathway may be a possible mediator for increased β-catenin, PI3K/Akt is also well known to cause accumulation of β-catenin through inactivation of GSK3β [173]. The nuclear accumulation of β-catenin correlates with tumor progression in cervical cancer patients [174]. Xuan et al [175] observed that the hedgehog-signaling pathway was also extensively activated in carcinoma and CIN of uterine cervix. Additionally, they reported that expression of the hedgehog-signaling pathway is greatly enhanced over the CIN I/II/III-carcinoma sequence in the uterine cervix. They suggested that the inappropriate activation of the hedgehog-signaling pathway and inactivation of p53 by E6 proteins from HR-HPV exert a synergistic effect on the uterine cervix carcinogenesis.

The Notch signalling pathway, which is necessary for several biological processes such as cellular proliferation, differentiation and apoptosis is considered an oncogenic pathway [169]. Recently, the product of the Notch1 gene has been identified as a novel target of p53. In cervical cancer, E6 can down-regulate expression of Notch1 through inactivation of p53. Therefore, its down regulation through p53 with E6/E6AP has been revealed as a novel tumor suppressor mechanism blocking development of HPV-induced cervical carcinogenesis [176]. The ErbB2 protein expression level is also regulated by p53 degradation and interference with this by E6/E6AP complexes contributes to cervical carcinogenesis [177]. The activation and deregulation of Notch signalling may provide a permissive environment for development of early pre-cancerous lesions which may lead to proliferation of HR-HPV associated cervical tumors.

Both E6 and E7 can deregulate cellular microRNA expression, which can alter cellular signaling pathways. Studies have shown that many miRNAs are involved in E6 and E7 mediated signaling pathways [178]. Aberrant expression of miRNAs has been reported to play a vital role in the progression of cervical cancer. Thus, a co-ordinated interaction of various pathways involving proteins and other biomolecules contributes towards progression to cervical carcinogenesis.

### Therapeutic strategies for improving HPV-mediated tumorigenesis of cervical cancer

#### Prophylactic vaccines

HPV prophylactic vaccine was a major breakthrough for cervical cancer prevention. Gardasil was the first quadrivalent cancer vaccine approved by the U.S. Food and Drug Administration in 2006 for prevention of cervical cancer, precancerous genital lesions, and genital warts caused by HPV6, HPV11, HPV16, and HPV18 [179]. Thereafter Gardasil®9, a nonavalent HPV-6/11/16/18/31/33/45/52/58 vaccine was approved. In 2009, Cervarix, bivalent vaccine was approved by FDA to prevent cervical cancer and precancerous lesions caused by human papillomavirus (HPV) types 16 and 18. These three vaccines effectively prevented HPV infections caused by the targeted types by eliciting the production of neutralizing antibodies that block the entrance of viral particles into host cells [180]. However, these vaccines were not effective at eliminating pre-existing infections, since the target antigens, L1 capsid proteins, are not expressed in infected basal epithelial cells [181]. A large number of individuals already infected with HPV did not benefit from these vaccines. In a clinical trial with 440 cancer patients, Rosenberg et al [182] reported that the objective response rate was low (2.6%) with a lack of powerful adjuvants capable of overcoming the immunosuppression present in cancer patients indicating that adjuvants are required to induce potent and durable immune response.

#### TLRs as vaccine adjuvants

At present, research and development of novel vaccine adjuvants are mainly focused on TLR ligands. Targeting TLR signaling pathways has been applied in clinical practice to improve the immunogenicity of DNA vaccines and promote the adjustment of T cells in resisting viral infection or to inhibit the wide spread inflammatory response caused by bacterial infection [183]. Investigations showed that simultaneous activation of multiple pathways of TLRs by vaccines resulted in better immunogenicity effects. Presently, only three TLR agonists are approved by international regulatory agencies for use in cancer patients: monophosphoryl lipid A (MPL), [184] bacillus Calmette-Guérin (BCG), and imiquimod [185]. Similar to LPS, MPL can activate the TRAM and TRIF signalling pathways and also can reduce the MYD-88 dependent signal pathway significantly that promoting inflammation [184]. Clinical trials using CpG ODNs as immunotherapeutic agents in cancer patients suggested that CpG ODN as monotherapy or in combination with chemotherapy can induce potent anti-tumor immune responses that correlate with clinical benefit [186]. Adjuvant systems using different combinations of TLR adjuvants, including alum, MPL, and CpG ODN, have shown better efficacy compared with a single TLR adjuvant [187]. TLRs as molecular adjuvants provide a new target for HPV infection prevention and provide direction for development of efficient vaccines.

#### Strategies targeting E6 E7 proteins

Several strategies that target E6 or the E6/E6-AP complex have been developed, including various therapies that employ cytotoxic drugs, a zinc-ejecting inhibitor of the viral E6 oncoprotein, an E6-AP mimetic epitope peptide (mimotope), an anti-E6 ribozyme, peptide aptamers that target the viral E6 oncoprotein, siRNAs that target the viral E6 oncogene, and combinations of therapies [188, 189]. Recent reports suggest a new strategy to induce viral E6 and E7 instability by using HSP90 and GRP78 inhibitors for the treatment of cervical cancer [190]. An E7 antagonist peptide showed antitumor effects through pRb reactivation both in vitro and in vivo [191]. GS-9191, a nucleotide analog prodrug showed an antiproliferative effect in vitro, and its topical application reduced the size of papillomas in the rabbit papillomavirus model [192]. Chitosan hydrogel containing granulocyte-macrophage colony-stimulating factor (GM-CSF) in combination with anticancer drugs showed antitumor effects through CD8+ T cell immunity [193]. Heparin-like glycosaminoglycans have been demonstrated to inhibit tumor growth by downregulation of HPV18 long control region activity in transgenic mice [194]. Finally, 5-aza-2′-deoxycytidine, a demethylating agent, and 5,6-dimethyl xanthenone-4-acetic acid, a vascular disrupting agent, in combination with therapeutic HPV DNA vaccines [195], showed significant antitumor therapeutic effects in vivo.

Furthermore, several plant-derived compounds have been investigated for their therapeutic potential in cervical cancer. In clinical trials, Praneem, a polyherbal formulation, was shown to eliminate HPV16 infection in early cervical intraepithelial lesions [196]. Curcumin, withaferin A, and epigallocatechingallate (EGCG), methyl jasmonate, also showed therapeutic effects via repression of viral oncogenes, upregulation of tumor suppressor genes, or induction of apoptosis in vitro [197, 198]. Withaferin A treatment in xenograft model showed significant reduction in tumor volume. Another natural compound, jaceosidin inhibited the functions of E6 and E7 oncoproteins in HPV16-positive cervical cancer cells [199].

#### RNAi-based Therapeutics against HPV

Recently, novel antiviral RNAi therapies have been developed and tested in clinical trials with short interfering RNAs (siRNAs) [200]. siRNAs are capable of selective silencing of endogenous genes in mammalian cells [201], and silencing viral genes in virus-induced diseases [202]. The RNAi targeting of E7 or E6/E7 led to the accumulation of TP53 and/or pRb, leading to induction of apoptosis and/or senescence in HPV16-positive cervical cancer cell lines, and in HPV18-positive human cervical cancer cells [203]. Zhou et al reported that two siRNAs targeting the E6/E7 promoter and E7 transcripts produced E6 and E7 mRNA knockdown, increased TP53 protein levels, decreased CDKN2A (p16INK4A) protein levels, and exhibited SiHa cell growth inhibition via apoptosis [204]. Another study reported that, HPV16 E6/E7 silencing by promoter-targeting siRNA was related to histone modification associated with histone H3-Lys9 methylation [205]. Chang et al [206] demonstrated that intratumoral administration of potent siRNA resulted in inhibition of tumor growth and induction of apoptosis in vivo, suggesting that siRNA treatment shows potential as an adjuvant therapy for cervical cancer.

#### Strategies Targeting Activation of TP53 Pathway

Another pathway that is often disrupted in cervical cancer is the TP53 pathway. Functional restoration of WT-TP53 may induce the regression of cervical carcinomas, which can be achieved by abrogating the expression of the E6 or E6/E7 oncogenes, or through cisplatin (cis-diaminedichloroplatinum II; CDDP) or radiation treatment. It has been demonstrated that, cisplatin therapy allows TP53 to escape from E6-mediated degradation, thereby facilitating TP53 accumulation in the nucleoli of HeLa cells [207]. Putral et al [208] investigated CDDP co-therapy, and found that shRNAs to E6 increased CDDP sensitivity in HeLa cells. Another recent study revealed that, intratumoral injection of both exonic (E6/E7-Exon) and intronic (E6/E7-Intron) siRNAs co-administration with intravenous injection of paclitaxel treatment restored the tumor-suppressive effect [209].

While both radiation therapy and chemotherapy have been used as treatment modalities in cancer patients, the advantages of combined chemo-radiotherapy have recently been reported. Cisplatin (cis-diaminedichloroplatinum II, CDDP) in combination with concurrent radiation is recommended for patients with disease at stage IIB or greater, and for those with locally advanced cervical cancer. Recently, it was demonstrated that TP53 showed expression in a wavelike or “pulsed” manner following exposure to ionizing radiation alone [210]. In addition, activation of the tumor suppressor pRb is part of the mode of action of HPV E6/E7 siRNA. Thus, complete reactivation of TP53 is possible, and its dynamics can be sustained by combination therapy with CCRT and HPV E6/E7 siRNA.

#### Epigenetic therapies

Epigenetic alterations, unlike genetic mutations, may be reversed by inhibiting the associated enzymes, and need to be evaluated as therapeutic modalities for HPV-associated lesions and cancers. Currently, two main classes of epigenetic drugs, methylation inhibitors and HDAC inhibitors, are in clinical trials for the treatment of cancer. Phase I study of Hydralazine in cervical cancer patients showed that different doses of hydralazine treatment was well-tolerated and effective to demethylate and reactivate the expression of eight tumor suppressor genes without affecting global DNA methylation [211]. Trichosanthin (TCS), a bioactive component isolated from a Chinese medicinal herb has been shown to have the capacity of restoring the expression of methylation-silenced tumor suppressor genes [212]. Valproic acid (VPA), an effective inhibitor of histone deacetylases, has been shown to modulate multiple cellular pathways including cell cycle arrest, apoptosis, angiogenesis, metastasis. The antitumor effect of VPA in cervical cancer may be caused due to either hyperacetylation of p53 protein protecting it from degradation by E6 and increasing p53 activity or via inhibition of Akt1 and Akt2 gene expression which resulted in Akt deactivation and apoptotic cell death [213]. Apicidin, a cyclic peptide HDAC inhibitor, was found to selectively downregulate DNA methyltransferase 1 [214] whereas trichostatin A (TSA), a classical HDAC inhibitor, was shown to inhibit DNA methyltransferase 3A [215]. In addition, the HDAC inhibitor suberoylanilide hydroxamic acid (SAHA) synergistically induces apoptosis in HeLa cervical cancer cells with bortezomib by activating caspase-3 and increasing the ratio of bax/bcl-2 expression [216]. Strategies targeting epigenetic aberrations appear promising therapeutic modalities for regulating cervical carcinogenesis.

## Conclusion and Perspectives

We have briefly seen in this mini review that multiple processes and signalling pathways contribute towards progression to oncogenesis. The primary viral factors responsible for altering these pathways and mediating progression to malignancy are the E6 and E7 proteins. The viral oncoproteins directly or indirectly trigger the deregulation of many control mechanisms that ultimately lead to the accumulation of genetic and epigenetic alterations. Recent studies have identified other equally important cellular targets, including telomerase, members of the DNA damage pathway, caspases and micro RNAs. Among these affected processes, genomic instability plays a central role leading to mutations in cellular genes which co-operate with tumor suppressor pathways leading to transformation and malignant progression.

The current HPV vaccination strategy targets at preventing the infection of few restricted HPV genotypes in uninfected individuals. They however have no effect on the existing HPV lesions and cancers. Women diagnosed with invasive and metastatic cervical cancer are in critical need of prognostic markers, targeted therapeutic options, and accurate surveillance strategies. Since it takes years to decades for cervical cancer development following acquisition of HPV infection, it provides us with a unique opportunity for cancer interception. Our understanding of the etiology of HPV-mediated carcinogenesis, the cellular pathways and molecular mechanisms involved in the transition from infection to cancer could provide novel opportunities for the design of effective therapeutic strategies to reduce the risk of HPV-mediated cancer.

## Abbreviations

Akt: serine/threonine-specific protein kinase
AP-1: Activator protein 1
Bcl-2: B-cell lymphoma 2
BRD4: Bromodomain-containing protein 4
CADM1: Cell adhesion molecule 1
CARM1: Coactivator-associated arginine methyltransferase 1
CBP: CREB-binding protein
CCNA1: Cyclin A1
CDH1: Cadherin 1
CDK 4: Cyclin-dependent kinase 4
CHK1: Checkpoint kinase 1
c-Myc: Proto-oncogene
CpG: Cytosine phosphate Guanine
CR1: Complement receptor 1
CYLD: Cylindromatosis Tumor Suppressor Protein Deubiquitinase
Cys: Cysteine
DAPK1: Death-associated protein kinase 1
DNA-PK: DNA-dependent serine/threonine protein kinase
DNMT1 DNMT3A and 3B: DNA methyltransferases 1, 3A, 3B
E1, E2, E4, E5, E6 and E7: Papillomavirus genome consisting of Early region (E) encoding six open reading frames
E2F: E2 factor family of transcription factors
E6AP: E6 associated protein
E6TP: E6 targeted protein
EDD: E3 Ubiquitin ligase
EMT: Epithelial-mesenchymal transition
EPB41L3: Erythrocyte membrane protein band 4.1 like 3
ERC55: Endoplasmic reticulum calcium-binding protein
FADD: Fas associated death domain protein
FIGO: Federation of Gynecology and Obstetrics
GAS5: Growth arrest-specific transcript 5
HDAC: Histone deacetylases
hDlg1: Disc large homolog 1
HMT: Histone methyltransferases
HOTAIR: Hox transcript antisense intergenic lncRNA
HR E6: High-risk E6
hTERT: Human telomerase reverse transcriptase
IARC: International Agency for Research on Cancer
IRF3: Interferon Regulatory Factor 3
L1: major and L2: minor capsid proteins
LCR: long control region
lncRNA-LET: lncRNA low expression in tumor
lncRNAs: Long non coding RNAs
MAGI1: Membrane associated guanylate kinase
MAL: Myelin and lymphocyte
MAPK: Mitogen activated protein kinase
MET: Mesenchymal Epithelial Transition
miRNAs: microRNAs
MMP-9: Matrix metallopeptidase 9
MPL: Monophosphoryl lipid
mTORC: mammalian target of rapamycin complex
ncRNA: Non-coding RNA
NFX1-91: splice variant of Nuclear transcription factor, X-box binding 1
NF-κB: Nuclear factor kappa B
NLS: Nuclear localization signals
NuRD: Nucleosome remodeling deacetylase
ORF: Open reading frame
p53: Tumor protein p53
PAX1: Paired box 1
PKC: Protein kinase C
pRb: Retinoblastoma protein
PRDM14: PR domain containing 14
PRMT: Protein Arginine Methyl Transferases
PSD95: Post synaptic density protein
PTEN: Phosphate and tensin homolog
RASSF1: Ras association domain family member 1
SAP97: Synaptic glutamate receptor dynamics
SET7: SET domain-containing protein 7
Snail: Zinc finger protein SNAI1
STAT: Signal transducer and activator of transcription
SV40: Simian virus 40
TLR: Toll-like receptors
TNFR1: Tumor necrosis factor receptor 1
TUSC8: TUSC8 tumor suppressor candidate 8
UBE3A: Ubiquitin-protein ligase E3A
UBR4: Ubiquitin protein ligase E3 component N- Recognin 4
VEGF: Vascular Endothelial Growth Factor
VIM: Vimentin
Wnt: Wingless-related integration site
ZO-1: Zonula Occludens 1
